RETRACTED

# RPN2 promotes metastasis of hepatocellular carcinoma cell and inhibits autophagy via STAT3 and NF-κB pathways

**DOI:** 10.18632/aging.102167

**Published:** 2019-09-03

**Authors:** Linsheng Huang, Zhiyuan Jian, Yi Gao, Ping Zhou, Gan Zhang, Bin Jiang, Yi Lv

**Affiliations:** 1 National Local Joint Engineering Research Center for Precision Surgery and Regenerative Medicine, Xi’an, Shaanxi Province, China; 2 Department of Hepatopancreatobiliary Surgery, Taihe Hospital, Hubei University of Medicine, Shiyan, Hubei Province, China; 3 The First General Surgery Department of the Hospital Affiliated Guilin Medical University, Guilin, Guangxi Province, China; 4 Department of Hepatobiliary Surgery, The First Affiliated Hospital, Xi’an Jiaotong University, Xi’an, Shaanxi Province, China

**Keywords:** RPN2, HCC, EMT, MMP-9, STAT3

## Abstract

This study aimed to investigate the function and the molecular mechanism of Ribophorin II (RPN2) in regulating Hepatocellular carcinoma (HCC) cell growth, metastasis, and autophagy. Quantitative real-time PCR (qPCR), western blotting analysis, and immunofluorescence assay were utilized to detect the RPN2 expression in HCC cell lines and specimens of HCC patients. We discovered that RPN2 expression was upregulated in HCC cell lines and tissues of HCC patients, which correlated with the low histological grade and low survival rate. Enhanced RPN2 expression stimulated cell proliferation, metastasis, invasion, and epithelial-mesenchymal transition (EMT), and decreased Microtubule-associated protein light chain 3B (LC3B) synthesis and reduced the expression of p62 protein. Further studies suggested that matrix metalloproteinase 9 (MMP-9) was partially upregulated by RPN2 via Nuclear factor kappa-light-chain-enhancer of activated B cells (NF-κB) p65. Interestingly, we found that phosphorylated RPN2 activated the signal transducer and activator of transcription 3 (STAT3) in HCC cells. It was also accountable for RPN2-stimulated elevated expression of MMP-9 and for invading HCC cells. It can be concluded that over-expression of RPN2 in HCC aggravated the malignant progression into cancerous cells. This research provided new evidences that RPN2 could facilitate tumor invasion by increasing the expression of MMP-9 in HCC cells.

## INTRODUCTION

Hepatocellular carcinoma (HCC) ranks among the top 10 cancers worldwide, with regard to prevalence and mortality [1]. It is a malignancy featured by poor prognosis and distant metastasis [2, 3]. Although there has been accumulating research concerning invasion and migration, the metastatic property of tumor remains the leading cause of death for patients with HCC and other tumors [4–8]. Even though there is substantial advancement in its diagnostic process and treatment, the mortality rate has remained considerably high in the last 5 years. Therefore, there is an imperative need to investigate and understand the innate mechanism that dictates metastatic behavior in HCC cells.

RETRACTED

According to clinical records, the high invasive ability of cancer cells is usually associated with poorer survival, suggestive of the aggravating contribution of strong invasive capability in the malignant development of cancer [9, 10]. In HCC, the macrophagocyte observed inside primary neoplasms is a general indicator of tumor progression and metastasis [11–14]. Macrophagocytes, after activation, are critical for the development and invasive process of tumors as they selectively up-regulate matrix-metalloproteinases (MMPs), which disrupt the extracellular matrix (ECM) and undermine basement membrane [15].

The highly conserved glycoprotein RPN2 exists only in rough endoplasmic reticulum (RER) membranes and participates in the translocation of secretory proteins and maintenance of the intrinsic uniqueness of the RER [16, 17]. Early studies have indicated that the oligo-saccharyl-transferase complex contains RPN2 protein and conjugates oligosaccharides and asparagine residues in the N-X-S/T common motif of the polypeptide strand [18, 19]. Moreover, previous studies have shown the suppressive effect of RPN2 depletion on the multiplication of tumor cells in osteosarcoma [20] and non-small cell lung cancer [21, 22]. Suppression of RPN2 was observed to be able to inhibit malignant breast tumors by inhibiting glycosylation of CD63 [23], which is a glycoprotein at the cell surface controlling cell mobility and invasiveness, as well as metastasis [24]. Similarly, the down-regulation of RPN2 triggered docetaxel-dependent programmed cell death and inhibited cell proliferation in the case of breast carcinoma by inhibiting glycosylation of the P-glycoprotein via N-glycosylation, and disrupting its membrane localization [25]. All the aforementioned studies indicated the significance of RPN2 as a mediator of N-linked glycosylation in both normal and drug-fast carcinoma cells. Comprehensive transcriptional recording and genome evaluations have shown that RPN2 could be a possible biological marker for colorectal cancer (CRC) cases [26].

Despite all the studies, the interrelation between RPN2 and HCC development, together with its underlying functional principles, remains obscure. Here, we aimed to investigate the effect of RPN2 on HCC development by employing various techniques. Collectively, through the use of western blotting (WB), real-time PCR (qPCR), and other methods, increased RPN2 expression was observed in HCC cells, and tumor tissue from human patients. The overexpression and silencing of RPN2 caused various effects on proliferation, migration, and invasion of HCC cells, and consequently affected the epithelial–mesenchymal transition (EMT) and autophagy. We also confirmed that RPN2 influenced HCC cell behavior by targeting STAT3 and NF-κB signaling.

RETRACTED

## RESULTS

### RPN2 level is increased in HCC cells and tissue specimens of HCC patients

Expression of RPN2 is relevant for the prognosis and diagnosis of different cancers. In the current research, when RPN2 gene expression was determined in HCC specimens vs normal healthy hepatic tissue, it was found to be significantly upregulated in the HCC specimens, compared to the normal healthy tissue (Figure 1A). Then, the mRNA levels of RPN2 in the human HCC cell lines, Huh-7 and HepG2 were compared with normal human hepatic cells (NHC) by qPCR. As shown in Figure 1B and 1C, mRNA levels of RPN2 were upregulated in HCC cells compared to the healthy cells. WB, performed to confirm the protein expression of RPN2 in the HCC cell lines and healthy cells, showed that the expression of RPN2 protein was considerably elevated in HCC cell lines, in comparison to the healthy hepatic cells (Figure 1D and 1E). In IFA imaging, more RPN2 staining was observed in Huh-7 and HepG2 than that in normal hepatic cells (Figure 1F and 1G).

**Figure 1:** **RPN2 expression in HCC cell lines and tissue specimens.** (**A**) RPN2 expression in specimens obtained from HCC patients (n = 20) vs normal healthy tissue (n = 20). (**B**, **C**) mRNA level of RPN2 in Huh-7 and HepG2 cells was determined by qPCR. (**D**, **E**) Protein expression of RPN2 in HCC cell lines, Huh-7and HepG2, as well as normal hepatic cells (NHC) was detected by WB. (**F**, **G**) Subcellular localization of RPN2 in HCC cell lines, Huh-7 and HepG2, was detected by immunofluorescence. RPN2 and nuclear DNA were stained with anti-RPN2 antibody (red) and DAPI (blue) respectively. Merged image showed the subcellular localization of RPN2. Images were captured on a fluorescence microscope. The band of target protein was normalized to the density of action. The quantification was performed independently in a single band. The experiments were performed three times. Results are recorded as mean ± SD. *P < 0.05, ***P < 0.001 vs control group**.**

### RPN2 mediates HCC cell proliferation

To confirm that RPN2 regulates the proliferation rate of HCC cells, the overexpression of RPN2 in Huh-7 and HepG2 cells was demonstrated with WB and qPCR (Figure 2A–2D). Further, MTT assay (Figure 2E and 2F) revealed that multiplication of Huh-7 and HepG2 cells, 12–72 h post-transfection, was greatly increased when they were transfected with RPN2-expressing adenovirus (AD-RPN2). The RPN2 overexpression caused a noticeable increase in colony numbers, evaluated by the soft agar colony formation assay, while transfection with the control (AD-NC) did not affect colony numbers of HepG2 cells (Figure 2G and 2H). To determine whether RPN2 overexpression promotes tumor phenotypes in normal hepatocytes, we performed RPN2 overexpression in normal hepatocytes (NHCs). However, there was no significant different in cell proliferation between RPN-overexpressing NHCs and control NHCs, indicating that RPN2 only exert its function in malignant cells (Figure 2I and 2J).

RETRACTED

**Figure 2:** **RPN2 overexpression promotes proliferation of Huh-7 and HepG2 cells.** The cell lines were transfected with AD-RPN2 and AD-NC (control). Western blotting (**A**, **B**) and qPCR (**C**, **D**) were conducted to confirm RPN2 overexpression in both the cell lines. (**E**, **F**) Multiplication of Huh-7 and HepG2 cells was measured at time points of 12, 24, 36, 48, 60, and 72 h after transfection by the MTT assay. (**G**, **H**) Soft agar colony formation assay of the Huh-7 and HepG2 cells expressing RPN2 and controls. (**I**) The NHC were transfected with AD-RPN2 and AD-NC (control). WB was conducted to confirm RPN2 overexpression in NHC. (**J**) Multiplication of NHC was measured at time points of 12, 24, 36, 48, 60, and 72 h after transfection by the MTT assay. The band of target protein was normalized to the density of action. The quantification was performed independently in a single band. The experiments were performed three times. Data are recorded as mean ± SD. **P <0.01 vs control group.

Previous research had reported that invasion and migration of HCC cells is a major cause of mortality during HCC development and progression [9]. To determine whether RPN2 influences the invasion and migration of HCC cells, transwell migration and wound-healing assays were carried out after transfection of HepG2 and Huh-7 cells with the RPN2-expressing adenovirus (AD-RPN2) and control (AD-NC). In the wound healing assay, overexpression of RPN2 promoted migration of Huh-7 and HepG2 cells towards the gap created by scratching of the cell monolayer (Figure 3A and 3B). Overexpression of RPN2 clearly increased migration of HCC cells (Figure 3C and 3D), especially in HepG2 cells, which is consistent with data from the wound healing assay. Moreover, we examined the effect of RPN2 overexpression on EMT; the ectopic expression RPN2 led to a decrease in E-cadherin and an increase in N-cadherin expression in both the cell lines, as determined by WB (Figure 3E and 3F). These data suggested that RPN2 overexpression facilitates the metastatic and invasive attribute of HCC cells *in vitro*.

RETRACTED

**Figure 3:** **Overexpression of RPN2 suppressed HCC cell migration and invasion.** After AD-RPN2 infection, migration and invasive process of HepG2 and Huh-7 cells were examined using injury healing (**A**, **B**) and transwell migration assays (**C**, **D**). (**E**, **F**) WB analysis was performed to examine E-cadherin and N-cadherin expression levels in HCC cells stably expressing RPN2. The band of target protein was normalized to the density of action. The quantification was performed independently in a single band. The experiments were performed three times. Data are recorded as mean ± SD. *P < 0.05, **P < 0.01 vs control group.

Next, the effect of RPN2 silencing in HepG2 and Huh-7 cells was determined by transfecting the cell lines with vector containing shRNA-RPN2 and control (vector containing shRNA), and then the gene and protein expression of RPN2 were determined by qPCR and WB (Figure 4A–4D). Cell proliferation was determined by MTT assay, and we found that RPN2 silencing caused a significant reduction in the number of HepG2 and Huh7 cells (Figure 4E and 4F). Additionally, colony formation assay showed a decrease in the number of colonies, compared to the control (Figure 4G and 4H).

**Figure 4:** **RPN2 silencing restrained HCC cell proliferation.** Western blotting (**A**, **B**) and qPCR (**C**, **D**) were conducted to confirm the silencing of RPN2 in both cell lines. (**E**, **F**) multiplication rate of Huh-7 and HepG2 cells was measured at the time points of 12, 24, 36, 48, 60, and 72 h after the transfection by using MTT assay. (**G**, **H**) Soft agar colony formation test was used to examine the replicative rate of HepG2 and Huh-7 cells transfected with shRNA-RPN2. The band of target protein was normalized to the density of action. The quantification was performed independently in a single band. Data are recorded as mean ± SD. *P < 0.05, **P < 0.01, ***P < 0.001 vs control group.

The effect of RPN2 silencing on the migration and invasion of HepG2 and Huh-7 cells was also determined by transwell migration and wound healing assays. The wound healing assay displayed that silencing of RPN2 inhibited the invasive capability of SMMC-7721 and HepG2 cells, compared to the control (Figure 5A and 5B). Further, RPN2 silencing remarkably reduced the number of migrated Huh-7 and HepG2 cells (Figure 5C and 5D), especially for HepG2 cells, which is consistent with wound healing data. Additionally, we examined the EMT-related protein expression upon RPN2 silencing. E-cadherin was significantly increased while N-cadherin was decreased due to RPN2 silencing (Figure 5E and 5F).

RETRACTED

**Figure 5:** **Silencing of RPN2 suppressed HCC cell migration and invasion.** After shRNA-RPN2 plasmid transfection, migration and invasive processes of HepG2 and Huh-7 cells were examined using injury healing (**A**, **B**) and transwell migration assays (**C**, **D**). (**E**, **F**) WB analysis detected the protein level of E-cadherin and N-cadherin in HCC cells transfected with shRNA-RPN2. The band of target protein was normalized to the density of action. The quantification was performed independently in a single band. Representative data from three separate experiments were recorded as mean ± SD. *P < 0.05.

### RPN2 regulates autophagy of HepG2 cells

It had been reported that RPN2 depletion induced autophagy via hypoxia signaling [27]. Therefore, our study looked at the effect of RPN2 overexpression and silencing on induction of autophagy in HCC cell lines. RPN2 overexpression did not significantly alter the autophagy rate of HepG2 cells, which was proved by the LC3B dynamic and processing (reduced LC3B I and II levels), but showed p62 upregulation (LC3B and p62, 2 main indicators of autophagic process [28]). On the contrary, RPN2 silencing induced a strong autophagy reaction: elevated LC3B IIlevel and (Figure 6A and 6B), and p62 degradation (Figure 6C and 6D). Quantitative PCR was also carried out to determine the p62 expression at mRNA level, and the results showed that its expression positively correlated with RPN2 expression (FIGURE 6E and 6F). Immuno-fluorescent assay was carried out to trace the location of LC3B protein upon RPN2 silencing. We observed that LC3B (green) gathered due to RPN2 silencing (Figure 6G). Electron microscopy was also performed to detect the autophagic vacuoles of cells with treatment to validate the autophagy state change. RPN2 silencing caused more autophagic vacuoles, when compared to the NCi groups (Figure 6H). These results demonstrated that RPN2 inhibited autophagy of HepG2 cells, which is partially responsible for its facilitative effect on proliferation of HCC cells.

**Figure 6:** **RPN2 depletion leads to autophagy.** Cells were firstly serum-starved for 24 hr. Then cells were treated with the solvent (DMSO) or 10 nM 3-Methyladenine (3-MA) for the indicated time before harvesting. (**A**, **B**) HepG2 cells were seeded onto 12-well plates, kept overnight and then starved for one day. Cells were infected with AD-RPN2 or transfected with shRNA-RPN2, and were serum-starved for 24 hr. Then cells were treated with the solvent (DMSO) or 10 nM 3-Methyladenine (3-MA) for the indicated time before harvesting. Whole cellular proteins were subjected to WB to indicate dynamic of LC3B Western blot analysis then determined the expression level of (**C**, **D**) p62 in cells with RPN2 overexpression and RPN2 silencing. (**E**, **F**) qPCR assay analyzed mRNA expression of p62 during RNP2 overexpression and silencing, respectively. (**G**) HepG2 cells were co-transfected with the shRNAs and GFP-LC3, as indicated, for 2 days. Cellular location of GFP-LC3B was then observed by IFA (magnification: 400x). (**H**) Autophagesomes were shown by transmission electron microscopy. Electron microscopy images of autophagic vacuoles in HepG2 and Huh-7 cells with silenced RPN2 or controls. Red arrows illustrate some of the autophagic vacuoles at different stages of the autophagy process (magnification: 2000x). The band of target protein was normalized to the density of action. The quantification was performed independently in a single band. The experiments were performed three times. Data were recorded as mean ± SD. **P <0.01, ***P <0.001 vs control group.

RETRACTED

### RPN2 induced MMP-9 expression through STAT3 and NF-κB pathways

It has been well-recognized that the invasive and metastatic nature of carcinoma cells were promoted, although partially, via generation of factors like MMP-9 [29]. Thus, we examined the expression of MMP-9 at both gene and protein level under varying RPN2 expression. We found that ectopic expression of RPN2 led to a drastic increasing of MMP-9 production (Figure 7A), while RPN2 silencing caused depletion of MMP-9 in HepG2 cell (Figure 7B). The qPCR data further confirmed that MMP-9 expression is positively correlated with RPN2 expression (Figure 7C and 7D). These data suggested that RPN2 played an essential role in MMP-9 expression in HepG2 cells.

**Figure 7:** **RPN2 regulated the MMP-9 expression level in the HCC cells.** HepG2 cells were transfected with AD-RPN2 or shRNA-RPN2. MMP-9 Protein and mRNA expression was detected via the WB (**A**, **B**) and qPCR (**C**, **D**). The band of target protein was normalized to the density of action. The quantification was performed independently in a single band. The experiments were performed three times. Data are represented as mean ± SD. **P <0.01 vs control group.

A previous study had shown that MMP-9 expression was modulated through STAT3 phosphorylation [30]; therefore, we next examined the STAT3 activation level with respect to RPN2 overexpression and silencing. As expected, the overexpression of RPN2 increased the phosphorylation level of STAT3 (Figure 8A) without affecting its expression, while RPN2 silencing remarkably reduced the phosphorylation level of STAT3 (Figure 8B). Furthermore, to confirm the effect of STAT3 in RPN2-induced MMP-9 upregulation, AG490 (an inhibitor binding to the upstream region of Janus kinase, the activating agent of STAT3) was utilized to block the signal transduction of STAT3 pathway. HepG2 cells stably expressing RPN2 were processed with 20 μM AG490 for 24 h. In response to AG490 treatment, STAT3 phosphorylation was clearly inhibited while its expression was not impaired. Meanwhile, MMP-9 expression was significantly reduced due to AG490 (Figure 8C). These evidences strongly indicated that STAT3 pathway was involved in the RPN2-regulated MMP-9 expression.

RETRACTED

**Figure 8:** **STAT3 is involved in RPN2-regulated MMP-9 expression level in HepG2 cells.** (**A**, **B**) HepG2 cells were transfected with AD-RPN2 or shRNA-RPN2 to modulate the expression of RPN2 expression. Protein expression and phosphorylation of MMP-9 and STAT3 was detected by WB. © HepG2 cells stably expressing RPN2 were treated with AG490 to block the STAT3 signal transduction. Protein expression of MMP-9 and STAT3 were then analyzed by WB. The band of target protein was normalized to the density of action. The quantification was performed independently in a single band. The experiments were performed three times. Data are represented as mean ± SD.

We then determined the function of NF-κB p65 in RPN2-induced MMP-9 production of HepG2 cells, as it is reported that the expression of NF-κB is related to the MMP-9 in different cell lines and diseases [31–33]. Therefore, we examined the p65 expression in HepG2 cells expressing RPN2. The expression of p65 and MMP-9 was significantly upregulated due to RPN2 overexpression (Figure 9A). In contrast, RPN2 silencing reduced p65 and MMP-9 level at protein level (Figure 9B). Moreover, qPCR data confirmed that p65 level is correlated with RPN2 expression (Figure 9C and 9D). In order to show the role of NF-κB p65 in RPN2-induced MMP-9 expression, NF-κB p65 expression was silenced with shRNA. The shRNA-p65 was transfected in HepG2 cell stably expressing RPN2, and the potency of transfection was further verified by WB. The p65 protein expression decreased in RPN2+shRNA-p65 group, due to which the MMP-9 expression was impaired, partially showing that NF-κB p65 regulated RPN2-induced expression of MMP-9 in HepG2 cells (Figure 9E).

**Figure 9:** **NF-κB is partially responsible for RPN2-mediated MMP-9 expressive level in HepG2 cells.** (**A**, **B**) HepG2 cells were transfected with AD-RPN2 or shRNA-RPN2 to modulate the RPN2 level, WB assay was conducted to examine the MMP-9 as well as NF-κB protein expression. (**C**, **D**) mRNA expression of MMP-9 and NF-κB p65 was then analyzed by qPCR. (**E**) HepG2 cells stably expressing RPN2 were transfected with shRNA-p65 to silencing the p65 expression. Protein expression of MMP-9 and p65 were then determined via WB. The band of target protein was normalized to the density of action. The quantification was performed independently in a single band. The experiments were performed three times. Data are represented as mean ± SD. *P < 0.05, ***P < 0.001 vs control group.

RETRACTED

## DISCUSSION

Mechanisms underlying the development of various tumors, such as HCC, are synergistic processes related to various gene transcriptions and signal transductions. Although previous studies have explored HCC, the understanding of the molecular mechanisms behind its development is currently insufficient. Some studies have reported that RPN2 is correlated with the development of various malignant tumor cells [20–23]; nevertheless, the exact working principles have yet to be studied and clarified. In a recent case, immunostaining of RPN2 protein demonstrated a remarkable connection with bad prognosis among CRC sufferers [26]. The current study demonstrated that RPN2, whose expression is increased in Huh-7 and HepG2 cell lines, and in the tumor tissue of HCC patients, plays an important role in the development and metastasis of HCC. Upregulation of RPN2 expression in the HCC cells enhanced cell proliferation, migration, invasion, and EMT; whereas the opposite was observed upon RNP2 downregulation. Further study has showed that RPN2 inhibited the autophagy of HepG2 cells, by augmenting LC3B processing and p62 degradation. Our data also suggested that RPN2 promoted the MMP-9 expression by mediating STAT3 phosphorylation and p65 expression. Autophagy is characterized by sequestration of bulk cytoplasm and organelles in double or multimembrane autophagic vesicles, and their delivery to and subsequent degradation by the cell’s own lysosomal system. Autophagy has multiple physiological functions in multicellular organisms, including protein degradation and organelle turnover. The recent implication of tumor suppressors like Beclin 1, DAP-kinase and PTEN in autophagic pathways indicates a causative role for autophagy deficiencies in cancer formation. Autophagic cell death induction by some anticancer agents underlines the potential utility of its induction as a new cancer treatment modality [34]. Our findings strongly suggest that RPN2 promoted HCC development via regulation of cell viability, migration, and autophagy by targeting the STAT3 activation and NF-κB p65 signaling, thus providing evidence that it is a potential agent for HCC therapy.

Proteases like MMP-9 are required for the invasion and destruction of extracellular matrix, thus boosting the invasive progression of cancerous cells to nearby healthy ones [35–37]. Increased expression of MMP-9 has been reported in head and neck squamous cell carcinoma (HNSCC) [36], and there is a positive correlation between MMP-9 expression and lymphatic metastasis [37] and laryngocarcinoma [38]. The current study showed that increased RPN2 expression in HCC samples was related to enhanced MMP-9 expression. As is known, MMP-9 from tumor and stromal cells, particularly macrophagocytes, has an indispensable position in the invasive, transferring, and angiogenic progression of malignant tumors. This study unveiled a new finding that RPN2 has an important function of elevating the MMP-9 expression in hepatic tumors by tyrosine phosphorylation of STAT3 signaling and enhanced NF-κB expression. For different malignant tumors, expression of p-STAT3 is closely associated with increased invasive and metastatic behavior among cancer cells [29]. Evidences suggested that activated STAT3 was involved in the process of MMP-9 expression and matrix degradation [39, 40], which enhanced the invasive capability of the drug-fast cancerous cells [35]. Our research demonstrated that activated STAT3, to some extent, could regulate RPN2-induced MMP-9 elevation in HepG2 cells. This is the first study to prove that STAT3-MMP-9 pathway could partly explain the RPN2-mediated invasive behavior of carcinoma cells.

RETRACTED

From the current data, we cannot exclude the possibility that our current findings caused by RPN2 overexpression or silencing is due to protein folding response in ER. A previous study has indicated that high expression of RPN2 resulted in increased glycosylation and altered cellular location of proteins in breast cancer cells, which could promote cancer malignancy. In contrast, inhibition of RPN2 expression reduced glycosylation, thereby attenuating cancer malignancy in breast cancer cells [23]. In Colorectal cancer (CRC) cells, decreased levels of MMP-2, MMP-9 and metastasis-associated protein 1, and increased levels of epithelial-cadherin and tissue inhibitor of metalloproteinases 2, were revealed in RPN2-upregulated cells [41]. Previous studies have also demonstrated that MMP-9 expression was positively-correlative with the phosphorylation of STAT3 and NFkB p65 [42, 43]. A previous study also suggested that phosphorylation levels of STAT3 and Janus kinase (JAK)2 were inhibited by RPN2 siRNA [44]. However, there is no report correlating p65 and RPN2. A schematic diagram has been provided to further elucidate the conceptual framework linking RPN2 function to a Stat3/NFkB/MMP-9 signaling pathway.

In several case, oncogenesis proceeds along with a temporary inhibition of autophagy. However, due to key role of autophagy in the preservation of intracellular homeostasis, autophagy commonly mediates oncosuppressive effects [45]. Accordingly, proteins with bona fide oncogenic potential inhibit autophagy, while many proteins that prevent malignant transformation stimulate autophagic responses [46]. In the present study, RPN2 downregulation caused autophagy of cells, which consequently impacted the viability and proliferation of cancer cells. Thus, the role of autophagy induced by RPN2 silencing in the present study is tumor suppressive.

RETRACTED

Overall, our study strongly suggested a multi-functional pro-tumor effect of RPN2 in the malignant properties of the two HCC cell lines, and that the development of HCC occurs via targeting both STAT3 and NF-κB. Nevertheless, we still cannot exclude other factors which RPN2 might target, and thus contribute to the HCC pathogenesis. Hence, more cross-talk assays need to be performed in future to screen and identify the targets for biotin-labeled RPN2 in HCC tissue specimens from patients and cell lines. In conclusion, this study provides evidence of a novel and important function of RPN2-mediated phosphorylation of STAT-3/p65 in the regulation of MMP-9 and cancer malignancy, including proliferation and invasiveness (Figure 10).

**Figure 10:** **Schematic model for the mechanism of RPN2-mediated STAT3/p65 phosphorylation pathway in HCC cells.** In HCC cells, RPN2 resulted in increased phosphorylation of STAT3/p65 and therefore enhanced transcription of MMP-9, which promoted cancer malignancy.

## MATERIALS AND METHODS

### Antibodies and chemicals

Antibodies for RPN2, STAT3, pSTAT3, p65, E-cadherin, N-cadherin, LC3B, p62, MMP-9, and Tubulin were purchased from Cell Signaling Technology (Danver, USA) and Santa Cruz Biotechnology (Dallas, USA), and Anti-HMGB1 antibody from GeneTex (Irvine, USA). The chemical AG490 was procured from Selleck (Beijing, China).

### Cells and transfection

Human cells Huh-7 and HepG2 were obtained from the Cell Bank of Academia Sinica (Shanghai, China), and cultivated in Dulbecco's modified Eagle's medium (DMEM; Gibco) supplemented with 10% fetal bovine serum, 2 mM L-glutamine, 100 μg/mL streptomycin and 100 U/mL penicillin. They were incubated at 37°C in a humidified atmosphere with 5% CO_2_. 5 × 10^6^ cells were seeded onto 6 and 12-well plates as per requirement and incubated overnight until 80–90% confluence.

### Clinical samples

The study group consisted of ten cases of HCC, with the age of the subjects ranging from 30–60 years. Clinicopathological data were obtained from the patients’ medical records. We harvested the para-neoplastic tissues at least one centimeter from the neoplastic tissues. All cases were hepatectomy candidates in the First Affiliated Hospital, Xi’an Jiaotong University. The study was approved by the Ethical Committee of the First Affiliated Hospital, Xi’an Jiaotong University. All study participants had given their written informed consent before participating in the study. Three pathologists reviewed and diagnosed the samples independently.

RETRACTED

### Adenovirus generation and transfection

The adenovirus was produced using the RAPAd^®^ CMV Adenoviral Bicistronic Expression System (Cell Biolabs, San Diego, USA) according to the manufacturer’s instructions. Human RPN2 cDNA was cloned into pacAd5 CMV-IRES linearized vector to form AD-RPN2. The purified linear DNAs were then co-transfected in 293T cells along with Lipofectamine™ 2000 reagent. Five days after the transfection, the adenoviruses were released from the 293T cells by performing the freezing-thawing procedure twice; the cell lysate was centrifuged to pellet the debris and the adenoviral lysate was stored at −80°C. For transfection of Huh-7 and HepG2 cells, 20 μL of AD-RPN2 from the adenoviral stock was used, and the cells were cultured for a period of 8 to 12 h. One adenovirus that expressed Green Fluorescent Protein (GFP) without RPN2 (AD-NC) served as the control.

### RNA interference

To reduce the expression of RPN2 and p65, short hairpin RNA (shRNA) against RPN2 and p65 were used. RPN2 and p65-targeted shRNA was designed and manufactured by Genomics Co., Beijing. The shRNA was added to 5 μL of RNase free water at a concentration of 100 pmol/μL, mixed with 10 μL transfection reagent, and kept for 15 min at 25 °C.

For the transfection assay, 5 × 10^6^ HCC cells Huh-7 and HEPG2 were seeded onto 6-well plates and incubated overnight at 37°C in 5% CO_2_ until 80-90% confluence, and then they were transfected with shRNA.

### MTT assessment

The MTT assay was performed to evaluate cell survival. Briefly, 20 μL of MTT (0.5 mg/mL) was added to the cells and incubated for 4 h at 37°C in an atmosphere of 5% CO_2_. The supernatant was discarded, 150 μL DMSO was added to each well, and rotated every 10 min to dissolve the purple formazan crystals. The absorbance was measured at 490 nm with an Infinite M200 microplate reader (Tecan, Männedorf, Switzerland).

### 3-Methyladenine (3-MA) treatment

For autophagy analysis, the cells have been pre-treated with 10 nM of 3-Methyladenine (3-MA), autophagy inhibitor. 3-M) is an inhibitor of phosphatidylinositol 3-kinases (PI3K). PI3K plays an important role in many biological processes, including controlling the activation of mTOR, a key regulator of autophagy. 3-MA inhibits autophagy by blocking autophagosome formation via the inhibition of class III PI3K [47].

RETRACTED

### WB

For the extraction of proteins, the cells were washed with PBS and then processed in RIPA Lysis Buffer (Cell Signaling Inc). Same volumes of total cellular proteins were separated with the SDS-PAGE, transferred onto the PVDF membrane, and immunoblotted with the commercial antibodies, as per requirement. Finally, the samples were immunoblotted with antibodies and treated as the control. For autophagy analysis, the cells have been pre-treated with 10 nM of 3-MA, autophagy inhibitor.

### Immuno-fluorescence assay (IFA)

For the LC3B puncta assay, the human prostate cancer cell line PC-3 was transfected with GFP-LC3B expression constructs (Addgene). Images were recorded under the fluorescent microscope as mentioned earlier [48]. The GFP puncta were calculated from 10 different microscopic fields. For autophagy analysis, the cells have been pre-treated with 10 nM of 3-MA, autophagy inhibitor.

### RNA extraction and qPCR

Trizol reagent was used to isolate total RNA from the cells. For, qPCR, the reaction mixture consisting of cDNA, forward and reverse primers and SYBR Green PCR Master Mix in a total volume of 20 μL was subjected to amplification in the Light-Cycler 480 Real Time PCR system (Roche, Basel, Switzerland) using the following program: 95°C for 10 min followed by 40 cycles at 95°C for 15 sec, 60°C for 30 s, and 72°C for 30 s. GAPDH was used as the internal reference. Quantification was performed according to 2^-ΔΔCT^ method through normalization to GAPDH. For autophagy analysis, the cells have been pre-treated with 10 nM of 3-Methyladenine (3-MA), autophagy inhibitor.

### Transwell migration assays

After 24 h transfection, the HCC cells were trypsinized, followed by washing with D-Hanks solution. Matrigel inserts (8 μm pore size) were used to separate the wells of a 24-well culture plate into top and bottom compartments. F-12 medium (400 μL) containing HGF (20 ng/mL) and FBS (10%) was added into the bottom chamber and the cells were seeded in the upper chamber. Following incubation, crystal violet was added to stain the cells that had migrated through the pore, and observed under a microscope (Zeiss).

### Wound healing assay

After 48 h of treatment, Cells (1 × 10^6^ cells/mL) were seeded in 24-well culture plate and grown until they reached 70–80% confluence. Using a sterile pipette tip, a scratch wound was created by scraping the monolayer of cells. The wells were washed twice with PBS to remove the detached cells, fresh medium was added and the cells were incubated for 0 (control) and 48 h. The cell images were obtained with an inverted microscope (Nikon).

### Statistical analysis

Results are represented as mean ± standard deviation (SD). Differences were analyzed using one-way ANOVA or Student’s *t*-tests. The threshold for significance was set at *P* < 0.05.
